This article has been retracted.

# Convallatoxin suppresses osteosarcoma cell proliferation, migration, invasion, and enhances osteogenic differentiation by downregulating parathyroid hormone receptor 1 (PTHR1) expression and inactivating Wnt/β-catenin pathway

**DOI:** 10.1080/21655979.2022.2080363

**Published:** 2022-05-29

**Authors:** Xin Liu, Ze Geng, Xiangyong Ding, Yan Lou, Xingquan Zhang

**Affiliations:** Department of Orthopaedics, Affiliated Hospital of Nanjing University of Chinese Medicine, Nanjing, Jiangsu, China

**Keywords:** Convallatoxin, osteosarcoma cells, malignant phenotype, osteogenic differentiation, PTHR1, wnt/β-catenin pathway

## Abstract

Osteosarcoma (OS) is the most common primary malignant bone tumor in children and adolescents. Convallatoxin, a natural cardiac glycoside, exhibits potent anti-tumor activities. Literature has confirmed that PTHR1 is highly expressed in OS tissues and cells and downregulation of PTHR1 could decrease the invasion and growth of OS cells and increase tumor differentiation. In addition, PTHR1 could activate Wnt signaling pathway to promote the malignant functions of OS. In the present study, MG63 and U2OS cells were treated with 0, 12.5, 25, and 50 nM convallatoxin in order to elucidate the precise function of convallatox on the malignant behaviors of OS cells. Moreover, MG63 and U2OS cells treated with convallatoxin were transfected with Ov-PTHR1 or sh-DKK1, aiming to explore whether convallatoxin impeded the malignant progression of OS by modulating PTHR1 and Wnt/β-catenin pathway. CCK-8, wound healing and transwell assays were employed to assess the proliferation, migration, and invasion of OS cells. Differentiation markers (collagen 1, osteopontin, RANKL, Runx2, osteocalcin) were measured to evaluate OS cell differentiation. Results illuminated that convallatoxin suppressed proliferation, migration, and invasion as well as promoted osteogenic differentiation of OS cells. Besides, convallatoxin inhibited PTHR1 expression and inactivated Wnt/β-catenin pathway and PTHR1 overexpression activated Wnt/β-catenin pathway. Furthermore, PTHR1 overexpression or DKK1 knockdown reversed the suppressing effects of convallatoxin on OS cell proliferation, migration, and invasion, as well as the enhancing effect of convallatoxin on OS cell osteogenic differentiation. Collectively, convallatoxin may repress the malignant progression of OS by blocking PTHR1 and Wnt/β-catenin pathway.

## Highlights

- Convallatoxin inhibits the malignant behaviors of OS cells.
- Convallatoxin increases osteogenic differentiation of OS cells.
- PTHR1 overexpression activates Wnt/β-catenin pathway.
- Convallatoxin represses OS progression by blocking PTHR1 and Wnt/β-catenin.
- Convallatoxin might be a promising medicine for OS therapies.

## Introduction

Osteosarcoma (OS), the most common malignant bone tumor, features high rates of metastasis and recurrence [1]. It is generally accepted that OS is a differentiation defect disease caused by genetic and epigenetic interference from the terminal differentiation of osteoblasts [2]. Recently, the rapidly increasing incidence and mortality of OS have become the main contributors to cancer death in children and adolescents [2]. Neoadjuvant chemotherapy combined with limb salvage surgery is the main therapy for OS, and the five-year survival rate can reach about 66–82% [3]. Nevertheless, as tumor progression comes as one of the main barriers in getting over OS, so that the five-year survival rate is only about 20% in patients with metastatic or recurrent disease [4]. In addition, rigorous problems, such as chemotherapy resistance and severe side effects limit the application of clinical chemotherapy drugs [5]. Hence, there is an urgent need to develop drugs with selective cytotoxicity to OS cells and to explore novel therapeutic targets against OS metastasis.

Cardiac glycoside, a class of steroidal glycosides with significant physiological activities, has been reported to possess potent antitumor efficacy and to selectively inhibit the proliferation of human tumor cells [6,7]. Convallatoxin, which can be found in lily of the valley (Convallaria majalis), is a natural cardiac glycoside [8]. Research has testified that convallatoxin exhibits obvious anti-tumor potential. Convallatoxin exerts desirable pro-apoptotic, anti-proliferative, and anti-angiogenesis effects on colorectal cancer cells [9,10]. Besides, convallatoxin shows dose- and time-dependent cytotoxic effects on breast cancer cells [11]. Nevertheless, the antineoplastic activity of convallatoxin on OS cells and the underlying molecular mechanisms have not been fully understood till now.

It has been reported that parathyroid hormone (PTH) and paracrine/autocrine PTH-related protein (PTHrP) are involved in tumorigenesis, bone development, and turnover [12,13]. As a common PTH/PTHrP receptor, parathyroid hormone receptor 1 (PTHR1) has been validated to be upregulated in OS tissues and cells [14]. Additionally, literature has confirmed that the knockdown of PTHR1 could decrease the invasion and growth of OS cells and increase tumor differentiation [15].

It is worth noting that PTHR1 could activate Wnt signaling pathway to promote the malignant functions of OS [16]. Wnt signaling pathway is a highly conserved pathway that regulates the development and homeostasis of many tissues [17]. Abnormal signals in Wnt signaling pathway are closely related to the occurrence of various cancers [18]. Research has verified that Wnt signaling pathway can participate in the development of OS [19].

Herein, the proliferation, migration, invasion, and osteogenic differentiation of OS cells were evaluated, so as to demonstrate the biological function of convallatoxin in OS pathological process. In addition, this designed work attempted to uncover the molecular mechanism underlying the protective effects of convallatoxin against the malignant progression of OS.

## Materials and methods

### Cell culture

Human OS cell lines (MG63 and U2OS) were obtained from American Type Culture Collection (ATCC, VA, USA) and cultured in high-glucose Dulbecco’s modified Eagle’s medium (HG-DMEM; Gibco, NY, USA) containing 10% fetal bovine serum (FBS), 100 U/ml penicillin, and 100 μg/ml streptomycin (Sigma-Aldrich, MO, USA) in a humidified atmosphere at 37°C with 5% CO_2_.

### Cell transfection

PTHR1 overexpression lentivirus (Ov-PTHR1), short hairpin RNA (shRNA) specific to DKK1 and their corresponding negative control (Ov-NC and sh-NC) were procured from GenePharma (Shanghai, China). In brief, MG63 and U2OS cells at a density of 4 × 10^4^ cells/well were seeded in 12-well plates and incubated until 90% confluence. The vectors and Lipofectamine 2000 reagent were separately incubated in serum-free Opti-MEM (Gibco, NY, USA) for 5 min and then mixed for an additional 20 min incubation. The mixture was added into cells, and cultured for 6 h. Next, serum-free medium was replaced with DMEM containing 10% FBS and cultured for 48 h. Cells were harvested for further analysis after 48 h transfection.

### Cell treatment

Convallatoxin (Sigma-Aldrich, MO, USA) was suspended in sterile water and stored at 4°C. MG63 and U2OS cells were treated with 0, 12.5, 25, 50, and 100 nM convallatoxin for 24 h.

### Cell counting kit-8 (CCK-8) assay

CCK-8 assay was adopted to measure the viability of MG63 and U2OS cells. The transfected or untransfeted cells were inoculated in 96-well plates at a density of 5 × 10^3^ cells/well. Following the designed convallatoxin treatment, 10 µl CCK-8 reagent (Beyotime, Shanghai, China) was added into each well and incubated for additional 4 h. The optical density (OD_450nm_) was measured using a microplate reader (Bio-Rad, CA, USA).

### Wound healing assay

Wound healing assay was adopted to assess the migrative abilities of MG63 and U2OS cells. MG63 and U2OS cells (1 × 10^6^ cells/well) were seeded into 6-well plate until 95% confluence. A ‘wound’ was created on the cell monolayer by utilizing sterile 200-µl pipette tips and the detached cells were then washed with PBS. Subsequently, cells were cultured in serum-free medium for 24 h. The wounded area was photographed and observed at 0 and 24 h under a microscope (magnification, ×100; Olympus, Tokyo, Japan) [20].

### Transwell assay

Transwell assay was adopted to assess the invasive abilities of MG63 and U2OS cells. MG63 and U2OS cells were re-suspended in serum-free medium and seeded at a density of 2 × 10^4^ cells/well into the upper compartment of 24-well transwell chambers (Corning, NY, USA) spreading with 50 µl of Matrigel (Solarbio, Beijing, China). Next, 600 µl medium containing 10% FBS was placed to the lower chamber. After 24 h incubation, noninvasive cells were gently removed and cells on the lower layer were fixed with 4% paraformaldehyde and stained with 0.1% crystal violet solution. The invaded cells were photographed and quantitatively counted under a microscope (magnification, ×100; Olympus, Tokyo, Japan).

### Western blotting analysis

Briefly, total proteins from MG63 and U2OS cells were isolated using radio-immunoprecipitation assay (RIPA) lysis buffer and protein concentration was quantified using a bicinchoninic acid (BCA) Protein Assay kit. Equal amount of protein samples (30 μg) were subjected to sodium dodecyl sulfate-polyacrylamide gel electrophoresis (SDS-PAGE) and then transferred onto polyvinylidene fluoride (PVDF) membranes. Nonspecific binding proteins were blocked with 5% nonfat milk, primary antibodies against MMP2 (Abcam, ab181286, 1:1000), MMP9 (Abcam, ab228402, 1:1000), Collagen 1 (Abcam, ab260043, 1:1000), osteopontin (Abcam, ab214050, 1:1000), RANKL (Abcam, ab65024, 1:1000), Runx2 (Abcam, ab23981, 1:1000), osteocalcin (Abcam, ab181286, 1:5000), DKK1 (Abcam, ab93017, 1:1000), β-catenin (Abcam, ab224803, 1:1000), PTHR1 (Abcam, ab189924, 1:1000), and GAPDH (Abcam, ab181602, 1:1000) were applied to incubate membranes overnight at 4°C. On the next day, secondary antibodies (Abcam, ab205718, 1:50,000) were employed to incubate membranes for 1.5 h at room temperature. Protein bands were developed with electrochemiluminescence (ECL) detection kit (Beyotime, Shanghai, China). Protein expression was analyzed using Image J software with GAPDH as the internal reference.

### Reverse transcription-quantitative polymerase chain reaction (RT-qPCR)

Total RNA was isolated from MG63 and U2OS cells using TRIzol reagent (Invitrogen, CA, USA). The complementary DNA (cDNA) was synthesized with PrimeScript RT Reagent Kit (Takara, Tokyo, Japan). Next, quantitative PCR analysis was carried out on an ABI 7500 system (Applied Biosystems, CA, USA) using SYBR Premix Ex Taq kit (TaKaRa, Tokyo, Japan). The PCR conditions were as follows: denaturation at 95°C for 20s, 40 cycles of denaturation at 95°C for 30s, annealing at 55°C for 30s and extension at 72°C for 30s. GAPDH served as the endogenous control. The primer sequences were listed as follows: PTHR1: forward 5'- CTCTTTGGCGTCCACTACATTG −3'; reverse 5'- TTGAGGAACCCATCGTCCTTG −3'; DKK1: forward 5'- ATAGCACCTTGGATGGGTATTCC −3'; reverse 5'- CTGATGACCGGAGACAAACAG −3'; GAPDH: forward 5'- CAGGAGGCATTG-CTGATGAT −3'; reverse 5'- GAAGGCTGGGG-CTCATTT −3'. 2^−∆∆Ct^ method [21] was applied to calculate the relative gene expression.

### Immunofluorescence staining

After fixation in 4% paraformaldehyde for 15 min, MG63 and U2OS cells were then permeabilized in 0.5% TritonX-100 solution. Following blocking in 5% BSA, primary antibody against collagen 1 was utilized to incubate cells overnight at 4°C. Next, fluorescent secondary antibody was employed to incubate cells for 1 h at room temperature and 4’, 6-diamidino-2-phenylindole (DAPI) was used to counterstain nuclei. Images were observed and photographed under a fluorescence microscope (magnification, ×200; Olympus, Tokyo, Japan).

### Statistical analysis

Data collected from three independent experiments were displayed as mean values ± standard deviation (SD). Comparisons among multiple groups were performed using one-way analysis of variance (ANOVA) followed by Tukey’s post hoc test. *P*< 0.05 indicates differences with statistical significance.

## Result

### Convallatoxin inhibits proliferation, migration, and invasion of OS cells

MG63 and U2OS cells were treated with 0, 12.5, 25, 50, and 100 nM convallatoxin for 24 h, aiming to explore the specific functions of convallatoxin on the malignant behaviors of OS cells. CCK-8 assay displayed that convallatoxin notably inhibited the viability of MG63 and U2OS cells in a dose-dependent manner Figure 1(a, b). Besides, results of wound healing and transwell assays indicated that convallatoxin dose dependently suppressed the migrative and invasive abilities of MG63 and U2OS cells Figure 1(c, d). MMP2 and MMP9 are gelatinases that are able to degrade and remodel ECM. For these reasons, MMP2 and MMP9 play important roles in promoting the metastasis of cells. Dose dependently reduced expressions of MMP2 and MMP9 in MG63 and U2OS cells treated with convallatoxin also suggested that convallatoxin could repress OS cell migration and invasion Figure 1(e, f).

**Figure 1.** Convallatoxin inhibits proliferation, migration and invasion of os cells. mg63 and u2os cells were treated with 0, 12.5, 25, 50 and 100 nm convallatoxin for 24 h. (a, b) cck-8 assay for determination of cell viability. (c, d) wound healing and transwell assays for determination of cell migration and invasion. (e, f) western blot assay for determination of mmp2 and mmp9 expressions. * *p* < 0.05, ** *p *< 0.01, *** *p* < 0.001 vs 0 nm convallatoxin.

### Convallatoxin increases osteogenic differentiation of OS cells

Herein, levels of differentiation markers (collagen 1, osteopontin, RANKL, Runx2, osteocalcin) were measured to evaluate OS cell differentiation. Dose-dependently increased protein expressions of collagen 1, osteopontin, Runx2, and osteocalcin and decreased RANKL protein expression were observed in MG63 and U2OS cells following convallatoxin treatment Figure 2(a, b). In addition, immunofluorescence staining also revealed that convallatoxin elevated collagen 1 level Figure 3(a, b). In a word, convallatoxin could promote osteogenic differentiation of OS cells.

**Figure 2.** Convallatoxin increases osteogenic differentiation of os cells. mg63 and u2os cells were treated with 0, 12.5, 25 and 50 nm convallatoxin for 24 h. (a, b) western blot assay for determination of collagen 1, osteopontin, rankl, runx2, osteocalcin expressions. * *p* < 0.05, ** *p *< 0.01, *** *p* < 0.001 vs 0 nm convallatoxin.

**Figure 3.** Convallatoxin increases osteogenic differentiation of os cells. mg63 and u2os cells were treated with 0, 12.5, 25 and 50 nm convallatoxin for 24 h. (a, b) immunofluorescence staining for determination of collagen 1 expression. * *p* < 0.05, *** *p* < 0.001 vs 0 nm convallatoxin.

### Convallatoxin suppresses PTHR1 expression and Wnt/β-catenin pathway

Additionally, convallatoxin reduced expressions of PTHR1 and β-catenin and elevated DKK1 expression in MG63 and U2OS cells in a dose-dependent manner Figure 4(a, b). These results indicated that convallatoxin could suppress PTHR1 and inactivated Wnt/β-catenin pathway in OS cells.

**Figure 4.** Convallatoxin suppresses pthr1 expression and Wnt/β-catenin pathway. mg63 and u2os cells were treated with 0, 12.5, 25 and 50 nm convallatoxin for 24 h. (a, b) western blot assay for determination of pthr1, dkk1 and β-catenin expressions. * *p* < 0.05, ** *p *< 0.01, *** *p* < 0.001 vs 0 nm convallatoxin.

### Overexpression of PTHR1 activates Wnt/β-catenin pathway

Furthermore, association between PTHR1 and Wnt/β-catenin pathway was investigated. Ov-PTHR1 was transfected into MG63 and U2OS cells to upregulate PTHR1 expression for functional experiments. The transfection efficiency was validated by performing RT-qPCR and PTHR1 expression was distinctly upregulated in MG63 and U2OS cells following transfection with Ov-PTHR1 Figure 5(a, b). Convallatoxin reduced PTHR1 expression in MG63 and U2OS cells, which was partially abolished by PTHR1 overexpression. Besides, upregulation of PTHR1 decreased DKK1 expression and increased β-catenin expression, reversing the suppressing impacts of convallatoxin on Wnt/β-catenin pathway Figure 5(c, d). To conclude, upregulation of PTHR1 could activate Wnt/β-catenin pathway in OS cells.

**Figure 5.** Overexpression of pthr1 activates Wnt/β-catenin pathway. (a, b) mg63 and u2os cells were transfected with ov-pthr1 or ov-nc. rt-qpcr for determination of pthr1 level. *** *p* < 0.001 vs ov-nc (c, d) mg63 and u2os cells treated with convallatoxin were transfected with ov-pthr1 or ov-nc. western blot assay for determination of pthr1, dkk1 and β-catenin expressions. *** *p* < 0.001 vs control, ^##^ *p* < 0.01, ^###^ *p* < 0.001 vs convallatoxin + ov-nc.

#### Convallatoxin inhibits proliferation, migration, and invasion of OS cells through suppressing PTHR1 expression and Wnt/β-catenin pathway

DKK1 is a known secretory Wnt/β-catenin inhibitor. Then, sh-DKK1 was transfected into MG63 and U2OS cells to downregulate DKK1 expression, ultimately leading to the activation of Wnt/β-catenin pathway Figure 6(a, b). Transfection with sh-DKK1 reduced DKK1 level in MG63 and U2OS cells, reversing the promoting effect of convallatoxin on DKK1 expression Figure 6(c, d). It was observed that the injured viability of MG63 and U2OS cells caused by convallatoxin treatment was partly recovered upon overexpression of PTHR1 or knockdown of DKK1 Figure 6(e, f). Besides, attenuated migrative and invasive properties as well as lowly expressed MMP2 and MMP9 in MG63 and U2OS cells treated with convallatoxin were partly recovered upon overexpression of PTHR1 or knockdown of DKK1 Figure 6(g, j). To sum up, convallatoxin may suppress the proliferative, migrative, and invasive abilities of OS cells by downregulating PTHR1 expression and inactivating Wnt/β-catenin pathway.

**Figure 6.** Convallatoxin inhibits proliferation, migration and invasion of os cells through suppressing pthr1 expression and Wnt/β-catenin pathway. (a, b) mg63 and u2os cells were transfected with sh-dkk1 or sh-nc. rt-qpcr for determination of dkk1 level. *** *p* < 0.001 vs sh-nc (c, d) mg63 and u2os cells treated with convallatoxin were transfected with sh-dkk1 or sh-nc. western blot assay for determination of dkk1 expression. *** *p* < 0.001 vs control, ^#^ *p* < 0.05 vs convallatoxin + sh-nc (e, f) mg63 and u2os cells treated with convallatoxin were transfected with ov-Pthr1 or sh-dkk1. cck-8 assay for determination of cell viability. (g, h) mg63 and u2os cells treated with convallatoxin were transfected with ov-PTHR1 or sh-dkk1. wound healing and transwell assays for determination of cell migration and invasion. (i, j) mg63 and u2os cells treated with convallatoxin were transfected with ov-pthr1 or sh-dkk1. western blot assay for determination of mmp2 and mmp9 expressions. *** *p* < 0.001 vs control, ^##^ *p* < 0.01, ^###^ *p* < 0.001 vs convallatoxin + ov-nc, ^δδ^ *p* < 0.01, ^δδδ^ *p* < 0.001 vs convallatoxin + sh-nc.

#### Convallatoxin increases osteogenic differentiation of OS cells through suppressing PTHR1 expression and Wnt/β-catenin pathway

Furthermore, whether convallatoxin could influence OS cell differentiation via regulating PTHR1 and Wnt/β-catenin pathway was explored. Increased protein expressions of collagen 1, osteopontin, Runx2 and osteocalcin as well as decreased RANKL protein expression in MG63 and U2OS cells treated with convallatoxin were reversed by overexpression of PTHR1 or knockdown of DKK1 Figure 7(a, b). Additionally, immunofluorescence staining also displayed that the enhancing impact of convallatoxin on collagen 1 expression was abrogated by overexpression of PTHR1 or knockdown of DKK1 Figure 8(a, b). Overall, convallatoxin may promote osteogenic differentiation of OS cells by downregulating PTHR1 expression and inactivating Wnt/β-catenin pathway.

**Figure 7.** Convallatoxin increases osteogenic differentiation of os cells through suppressing pthr1 expression and Wnt/β-catenin pathway. mg63 and u2os cells treated with convallatoxin were transfected with ov-PTHR1 or sh-dkk1. (a, b) western blot assay for determination of collagen 1, osteopontin, rankl, runx2, osteocalcin expressions. *** *p* < 0.001 vs control, ^##^ *p* < 0.01, ^###^ *p* < 0.001 vs convallatoxin + ov-nc, ^δ^ *p* < 0.05, ^δδ^ *p* < 0.01, ^δδδ^ *p* < 0.001 vs convallatoxin + sh-nc.

**Figure 8.** Convallatoxin increases osteogenic differentiation of os cells through suppressing PTHR1 expression and Wnt/β-catenin pathway. mg63 and u2os cells treated with convallatoxin were transfected with ov-PTHR1 or sh-dkk1. (a, b) immunofluorescence staining for determination of collagen 1 expression. *** *p* < 0.001 vs control, ^###^ *p* < 0.001 vs convallatoxin + ov-nc, ^δδδ^ *p* < 0.001 vs convallatoxin + sh-nc.

## Discussion

OS has emerged as a major health problem in children and adolescents. The occurrence of OS tends to be originated from the terminal differentiation of osteoid cells or the process of Bone Marrow Stromal cells (BMSCs) differentiating into osteoid cells [2]. At the same time, the early stage migration and local invasion abilities are also prominently developed, ultimately resulting in the death of OS patients [3,5]. As a consequence, there is a critical need to explore effective drugs or molecular targets that can availably arrest OS progression.

Over the years, convallatoxin has been recognized as a potential novel drug to treat malignant tumors due to its strong anti-cancer activity and chemotherapy sensitization effect [22]. Schneider et al. [5] have reported that convallatoxin exerts potent anti-proliferative, anti-migratory, and anti-invasive effects on lung cancer cells [23]. Kaushik et al. [11] have indicated that convallatoxin could suppress the migration and invasion of human ER^+^ and triple-negative breast cancer cells. Besides, Zhang et al. [9] have demonstrated that convallatoxin exhibits inhibitory effects on the proliferation, metastasis, and angiogenesis of colorectal cancer cells via crosstalk between mTOR/STAT3 and JAK/STAT3 pathways. In the present study, it was revealed that the proliferation, migration, and invasion of MG63 and U2OS cells were suppressed after convallatoxin treatment. It was noted that convallatoxin exhibited inhibitory effects on the biological behaviors of OS cells in a dose-dependent manner. Besides, convallatoxin could also promote osteogenic differentiation of OS cells. These results clearly demonstrated that convallatoxin could suppress the malignant progression of OS.

Not only that, previous study has verified that PTHR1 is markedly elevated in OS tissues and cells and highly expressed PTHR1 is related to greater risk of metastasis and a poor prognosis [14]. In addition, PTHR1, which is positively correlated with the expressions of MMP2 and MMP9 in OS, could trigger the proliferation, invasion, adhesion, and migration of OS cells [24,25]. Furthermore, literature has reported that PTHR1 could promote the malignant functions of OS by activating Wnt signaling pathway [16]. As an important molecule in intracellular signal transduction, Wnt signaling pathway participates in a series of cell behaviors, such as proliferation, migration, and angiopoiesis [17]. Additionally, research has confirmed that Wnt signaling pathway is a critical player in the initiation and development of OS, thus acting as a potential target for OS therapy [18]. In the current work, it was demonstrated that convallatoxin reduced PTHR1 expression and inactivated Wnt/β-catenin pathway in OS cells and upregulation of PTHR1 could activate Wnt/β-catenin pathway. Moreover, the injured viability, attenuated migrative, and invasive properties, as well as increased osteogenic differentiation of OS cells treated with convallatoxin were partially abolished by overexpression of PTHR1 or knockdown of DKK1.

## Conclusion

To conclude, this work testified that convallatoxin exhibited inhibitory effects on OS cell proliferation, migration, and invasion as well as exerted enhancing effect on OS cell osteogenic differentiation by downregulating PTHR1 expression and inactivating Wnt/β-catenin pathway. These findings prompted that convallatoxin might be a promising medicine for OS therapies clinically.

## Supplementary Material

Supplemental Material

## Data Availability

The analyzed data sets generated during the present study are available from the corresponding author on reasonable request.
